# Application of New Media in Student Management from the Perspective of Deep Learning and Evaluation and Analysis of Practical Effects

**DOI:** 10.1155/2022/1765448

**Published:** 2022-06-09

**Authors:** Danjun Ji, Xuejiao Wang, Tianyu Zhang

**Affiliations:** School of Literature and Journalism, Sanjiang University, Nanjing, Jiangsu 210012, China

## Abstract

New media has become incorporated into people's lives as a result of its advent and great popularity. Students make substantial use of new media, and using it for student management necessitates social attention and assistance. It has to do with the management effect of colleges and universities, as well as the development of college students and societal harmony and advancement. Under the new media environment, student management workers should apply new media to daily student management work on the basis of traditional student management work methods, carry out new extensions and expansions, and use various forms of new media platforms as working methods and means. To carry out student work to improve the efficiency and effectiveness of student management work, in this context, this paper uses deep learning to carry out the application and practical effect evaluation of new media in student management and completes the following work: (1) This paper examines and discusses the development history, concept, connotation, and characteristics of new media using the literature analysis approach. The literature is used to synthesize the study findings of contemporary academic circles on the management of student issues in the new media environment. (2) The related technologies of BPNN are introduced, the evaluation index of the application effect of new media on student management work is constructed, and then, the appropriate BPNN structure is designed. (3) Experiments are carried out with the self-designed data set. The results of the experiments reveal that the model proposed in this research has a low error and good performance.

## 1. Introduction

In this rapidly developing society of digital technology and new media technology, all kinds of media information have enriched people's information resources. The majority of young college students are one of the groups that use new media widely and have been integrated into the new media era [1]. How to use new media to serve student management and open up a new situation of new media platform education has become a new topic for student management workers in colleges and universities. There are now over 750 million Chinese netizens, 720 million mobile netizens, and more than 50 percent Internet penetration in China, according to a CNNIC report issued in August 2017 entitled “Statistics on the Internet Development in China.” In terms of age structure, Chinese netizens are mainly 10-39 years old, accounting for about 70% of the total, among which the 20-29 age group accounts for the highest proportion of netizens, close to 30. In terms of occupational structure, netizens have the largest group of middle school students, accounting for about 25%. Among the student groups of Chinese netizens, college students are one of the subjects who use new media. The emergence of new media has changed the way of information production and dissemination and has formed a variety of publicity media including Weibo, WeChat public account, and website, which has brought an impact on the management of college students [2]. For example, many colleges and universities still use traditional management methods, mainly relying on manpower management. But it is more of an opportunity. College students born in the Internet age have taken the Internet and new media as part of their lives and have completely accepted new media.

New media provides colleges and universities with a more efficient and convenient management method, which enables the dissemination of traditional media content information from chain-like dissemination to network dissemination, which speeds up the speed and breadth of information dissemination and expands the influence of information [3]. The management of students in colleges and universities should make full use of this information dissemination tool to realize the informatization of student management. It is practical and feasible to use new media for student management, and it has a certain material basis. At present, “post-90s” college students are the main body of contact and use of new media, and mobile phones and tablet computers are the main forms of new media, and these new media terminals are widely owned by college students and young teachers, especially college students' mobile phone ownership rate is very high, which lays a solid material foundation for the application of new media to student management [4]. To break through the restrictions of time and distance, the new media can be easily carried and used, and the costs of new media information transmission are cheap, paving the way for the use of new media in student management. According to the “Higher Education Law” of my nation, the purpose of higher education is to educate highly skilled specialists with a creative spirit and practical aptitude, to foster a culture of science and technology, and to advance socialist modernization [5]. Numerous educational institutions use new media in their everyday operations to better manage college students, and this has resulted in an increase in student management efficiency as well as an increase in the effectiveness of the methods they use. The emergence of new media has also made it more difficult for colleges and universities to govern their operations, and many institutions lack the backing of solid ideas and management practices [6]. This paper takes the management of college students as the research object and analyzes the relatively backward management mode in the new media environment.

It argues that current management is complicated by the management environment, that managers lack knowledge of new media management, that managers' authority has eroded, and that individual students are preoccupied with issues such as the network, and then proposes a path for innovative management, and then uses deep learning to evaluate the value of new media in student management work. Dissemination of information occurs quickly and over a broad spectrum in the new media environment. In order to effectively manage college students, a university student management system must incorporate new media, constantly innovate management concepts and methods, fully utilize new media, and correctly understand the characteristics, development laws, and trends of new media. Excellent student management is a must in the age of social media [7]. As a result, one of the most pressing concerns confronting today's student employees is how to make the best use of digital media in overseeing college students.

The paper's organization paragraph is as follows: The related work is presented in Section 2.  Section 3 analyzes the methods of the proposed work.  Section 4 discusses the experiments and results. Finally, in Section 5, the research work is concluded.

## 2. Related Work

Although the time from the emergence, development, and widespread application of new media is relatively short, it has already received widespread attention from the society. Domestic scholars engaged in new media research have already formed a lot of research results. Regarding the definition of the concept of new media, scholars differ in terms of understanding and interpretation. At present, the academic circle has not formed a relatively unified concept expression. Reference [8] explains the concept of new media from four aspects: first, new media should be digital and highly interactive; second, new media is changing with technological development; third, so-called new media should adopt international standards as the judgment criteria; fourth, terminals are used to access information and services provided by terminals in new media. Reference [9] believes that the concept of new media is constantly developing, and new media has different forms of expression in different time periods. There are two types of new media: broad and narrow. In the broad sense, “new media” refers to new forms of communication or media based on digital, network, and other technologies; in the restricted sense, “new media” refers to “developing media.” Compared with traditional media such as newspapers, TV, and radio, new media is a communication platform that provides users with information and services based on digital technology, using mobile communication channels such as the Internet, and using computers and mobile phones as terminals [10]. Regarding the research on the manifestations of new media, reference [11] believes that the manifestations of new media include teletext, optical fiber cable communication network, computer communication network, TV, mobile phone, large-scale computer database communication system, multimedia information interactive platform, satellite live TV system, Internet, and multimedia technology broadcasting. There has been much study done on the coupling of new media and higher education, with an emphasis on the influence of new media on college students' ideological and political education, and how to lead college students ideologically in the new media environment. Most of the research is still at the level of theoretical research, and there are very few researches that really apply and test new media in practical work. There is a lot of attention on two components of college student affairs management research.

On one side, it highlights and examines problems with college and university administration's student affairs policies. According to reference, traditional college student affairs management in our country has flaws with the system, concept, and team structure. College administrators should adopt the management philosophy of “people-oriented” so that students have greater possibilities to participate in school management. Provide students with a good campus environment, cultivate students' self-awareness, encourage students to start their own businesses, and provide students with a platform for free development. On the other hand, it studies the management mode of college students. Reference [12] proposed that colleges and universities should change the simple management method, add services to the traditional “education-management” model, and take “student development” as the core of student management. Research on new media and student affairs management. The rise and wide application of new media in China has been relatively short. In recent years, my country's new media technology has made great progress, but the systematic research on new media applications is in its infancy. Reference [13] analyzed the impact of new media on the management of student affairs in colleges and universities and summed up three ways that current college student affairs management workers treat new media: one is to resist some new media with bad information; tired of dealing with the negative information on the new media; and thirdly, only hope to release information through some functions of the new media.

Reference [14] analyzed the characteristics of new media and the impact of new media on college students and analyzed the student service mechanism, news release mechanism, opinion hearing mechanism, leadership reception mechanism, democratic evaluation mechanism, emergency handling mechanism, and network literacy. The establishment of management mechanism makes suggestions to colleges and universities. According to reference [15], new media will present chances and problems for college students' work. New media qualities such as immediacy, variety, and equal communication, for example, provide a new platform for the creation of working methods and student affairs management methods in colleges and universities. In the United States, student management work is called student affairs management, which is similar to the student management work in Chinese universities in terms of work object, nature, content, and scope [16]. Reference [17] defines student affairs as follows. Student affairs are used to describe the organizational units and machines that are responsible for students' extraclassroom education and also include in-classroom education. In the management of student affairs in western developed countries, especially in the higher education in the United States, there is already a relatively complete theoretical and practical system, and the enterprising spirit and open tradition have achieved the first-class education status of the United States. The United States is a multiethnic and multicultural country, and politically, it is a country of decentralization. In this context, the management of student affairs in American colleges and universities presents the characteristics of diversity and individuality. The United States comprehensively promotes the concept of student development, educating students and serving students at the same time, and has made a new interpretation of the connotation of higher education [18–20]. By combing the above literature, it is found that scholars have paid attention to the impact of new media on colleges and universities and have carried out relevant research on how to apply new media. Studies into how students' political and ideological perspectives are being shaped in the new media era have been quite methodical and thorough, resulting in a wealth of theoretically sound study findings

## 3. Method

In this section, we define the basic theory of BP neural network, evaluation of the application effect of new media in student management, and construction of the evaluation model in detail.

### 3.1. The Basic Theory of BP Neural Network

BPNN is one of many branches of neural network. As far as the current research situation at home and abroad, it is a relatively mature theory. The BPNN performs calculation and fitting on a large amount of data, and each calculation will modify the internal parameters to increase the overall fitting effect of the model, so that the output results continue to approach the real data. The general BPNN structure consists of three parts. The first part is the input layer, which is the input end of data import and is an *N*-dimensional vector; the second part is the hidden layer. The hidden layer can be a multilayer network, but the middle layer of the general one-layer structure is enough to fit any mapping relationship; the third part is the output layer, which is the mapping result of the input data, which is an *N*-dimensional vector. A simple neural network model with one layer in the middle is shown in Figure 1. In the network structure, the units of the same layer are not connected to each other, and the units of the adjacent layers have a transfer connection.

The mathematical model of the neuron unit is as follows:

(1) $$\begin{array}{c} y=f\left[\overset{n}{\underset{i=1}{\sum }}w_{i}x_{i}-\lambda \right], \end{array}$$

where *y* is the output value of the neuron in the backward direction, *w*_*i*_ is the connection weight coefficient between the neural unit in the front layer and the neural unit in the rear layer, ∑*w*_*i*_ is the weighted summation value, *λ* is the threshold set by the neural network, and *f* is the activation function of the neural unit. The backward output value ∑*w*_*i*_*x*_*i*_ adjusted by the weight coefficient is compared with the set threshold *λ*.

After meeting certain conditions, the neural unit will work; otherwise, it will remain static. This working mode is essentially the input data. Perform category filtering to obtain different expected output values for input values in different categories. In a neural network, information is passed backward through the input layer through connection weight adjustment, and the neuron is activated when the weighted sum value satisfies the threshold condition.

The BPNN goes through the forward propagation process and the back propagation algorithm. The neural network first randomly assigns adjustment coefficients to the forward pass between each level and then fits the data samples. According to the comparison error between the output result and the given result, the weights of each layer are adjusted in a specific direction from the first layer along the middle layer to the last layer until the error reaches an ideal level. This algorithm is the error back propagation algorithm, namely, BP algorithm, and its related theory is as follows. Because the three-layer neural network is enough to simulate any mapping relationship, it is assumed that there is a three-layer network, the number of units in the first layer is *m*, the number of units in the second layer is *z*, and the number of units in the last layer is *s*. *X*_1_, *X*_2_, ⋯, *X*_*m*_ are input data; *H*_1_, *H*_2_, ⋯, *H*_*z*_ are the back-transmission data of the intermediate layer; and *y*_1_, *y*_2_, ⋯, *y*_*s*_ are output data. The adjustment coefficient from the *m*-th first-layer unit to the *z*-th intermediate-layer unit is *w*_*mz*_, the threshold of the *z*-th unit in the intermediate layer is *θ*_*z*_, the adjustment coefficient from the *z*-th intermediate-layer unit to the *s*-th last-layer unit is *R*_*zs*_, and the last threshold of the *s*-th unit of the layer is *φ*_*s*_; the transfer function from the first layer to the middle layer is *f*_1_, and the transfer function from the middle layer to the last layer is *f*_2_. Here, tansig is selected as the transfer function for *f*_1_ and *f*_2_. The input of the *z*-th unit of the second layer can be obtained:

(2) $$\begin{array}{c} \text{Ne}{\text{t}}_{\text{in}1z}=\overset{m}{\underset{i=1}{\sum }}x_{i}∙w_{iz}. \end{array}$$

The output of the *z*-th unit of the second layer is as follows:

(3) $$\begin{array}{c} H_{z}=f_{1}\left[\text{Ne}{\text{t}}_{\text{in}1z}-\theta_{z}\right]. \end{array}$$

The input to the *s*-th unit of the last layer is as follows:

(4) $$\begin{array}{c} \text{Ne}{\text{t}}_{\text{in}2s}=\overset{z}{\underset{i=1}{\sum }}H_{i}∙R_{\text{is}}. \end{array}$$

The output of the *s*-th unit in the last layer is as follows:

(5) $$\begin{array}{c} Y_{s}=f_{2}\left[\text{Ne}{\text{t}}_{\text{in}2s}-\varphi_{s}\right]. \end{array}$$

The output of the neural network is

(6) $$\begin{array}{c} O_{s}=\left(Y_{1},Y_{2},\cdots Y_{s}\right). \end{array}$$

Calculate the error of the prediction result with the least square method:

(7) $$\begin{array}{c} E_{k}=\frac{1}{2}\overset{s}{\underset{i=1}{\sum }}{\left(Y_{i}-y_{i}\right)}^{2}. \end{array}$$

Now adjust the parameter value according to the obtained error to reduce *E*_*k*_ and improve the explanatory power of the model. Obtain the partial derivative for the parameter Param that needs to be adjusted, so that the parameter changes in the opposite direction of the positive and negative signs of the partial derivative. At this time, the value of each unit change of the parameter operation is *∂E*_*k*_/*∂*Param. At the same time, in order to prevent the change rate from being too fast to miss the optimal parameter setting or the solution speed that is too slow, a reasonable learning rate *α* needs to be set. The parameter adjustment formula at this time is

(8) $$\begin{array}{c} {\text{Param}}^{\prime }=\text{Param}-\alpha \frac{\partial E_{k}}{\partial \text{Param}}. \end{array}$$

The weight adjustment from the second layer to the last layer can be obtained accordingly:

(9) $$\begin{array}{c} R_{zs}^{\prime }=R_{zs}-\alpha \frac{\partial E_{k}}{\partial R_{zs}}. \end{array}$$

The adjustment coefficient correction value ∆*R*_*zs*_ from the *z*-th unit of the second layer to the *s*-th unit of the last layer is

(10) $$\begin{array}{c} {\Delta R}_{zs}=-\alpha \frac{\partial E_{k}}{\partial R_{zs}}=-\alpha \frac{\partial E_{k}}{\partial Y_{s}}∙\frac{\partial Y_{s}}{\partial \text{Ne}{\text{t}}_{\text{in}2s}}∙\frac{\partial \text{Ne}{\text{t}}_{\text{in}2s}}{\partial R_{zs}}. \end{array}$$

Of which there are

(11) $$\begin{array}{c} \frac{\partial E_{k}}{\partial Y_{s}}=Y_{s}-y_{s}. \end{array}$$

The above is the mathematical principle of the BP algorithm for parameter correction. Using the relevant network, generally only need to set the relevant index parameters, and then, the adjustment between the layers of the BPNN can be adjusted by fitting the abovementioned correction model with sufficient sample data. The coefficient is corrected and calculated, and the nonlinear mapping relationship between the input information and the output information is simulated and fitted.

### 3.2. Evaluation of the Application Effect of New Media in Student Management

#### 3.2.1. Diversified Types of New Media

The “Regulations on the Administration of Students in Ordinary Institutions of Higher Education” pointed out that the management of students is to maintain the normal order of education, teaching, and life in ordinary institutions of higher learning; protect the legitimate rights and interests of students; and cultivate socialist builders who develop in an all-round way in terms of morality, intelligence, physique, beauty, and successor. The supervision of college students is an important aspect of college administration. Because of the rapid increase of informatization and digitalization, students at colleges and universities are increasingly using mobile devices on campus, such as smartphones and tablet computers. New media is subtly changing the traditional management model of college students. Taking a university as an example, this paper investigates the current situation of using new media to carry out student management, the problems existing in the process of using new media for student management, and analyzes the reasons. The types of new media used are diversified. Currently, the more popular new media softwares include instant messaging software, video software, dating software, etc. The instant messaging software developed by Tencent is the most widely used, and QQ and WeChat are the most representative. Users can communicate instantly through mobile digital media by sending pictures, expressions, audio, video, etc. A whopping 889 million people use WeChat on a monthly basis as of December 2016. For chatting with pals, WeChat is a cutting-edge social networking app. Users can add friends and follow public platforms by searching WeChat, sharing WeChat, shaking, scanning QR code, etc., and can share with your friends by posting text, pictures, and videos in your moments. From the perspective of college student management, the WeChat platform, as a management tool, has been valued by many colleges and universities, and they have begun to use the WeChat platform to serve the management of students. We discovered through research and interviews that a certain school has begun to experiment with new media platforms to help with student management, and the sorts of use are becoming broader. The main forms of use include the establishment of theme education websites specially used for student management, such as the website of the Ministry of Student Affairs and the National Defense Education website. Different education systems also provide management services for college students through various forms such as QQ, WeChat, Weibo, and forums. Students' questionnaires can reflect this conclusion. In the interviews with teachers, the vast majority of teachers choose instant messaging tools and Weibo, post bar, forums, etc. These data show that colleges and universities have begun to use a variety of new media platforms to carry out student management work and have achieved certain results.

#### 3.2.2. Changes to Student Management by New Media

Through interviews and questionnaires, we learned that the student management work of a certain school is making continuous progress relying on new media platforms. The specific manifestations are as follows:

1. New media promotes the digitalization and networking of student management work. We have entered the digital age, and new media makes student management work to be digitalized and networked. In the past, in order to understand the basic situation of students, the collection of student information was in the form of a paper information registration form. The student information is now almost entirely computerized. Student information, namely, basic student information, rewards and punishments, mental health, employment, and so on, is all provided to the data platform of a digital campus of a particular school. When you need to access student information, you can utilize it to quickly search for digital data, making student management more efficient and eliminating the need for significant human labor. It simplifies a lot of repetitive work, saves manpower, reduces workload, avoids mistakes in some work, improves work efficiency, and expands the work extension space of student administrators
2. The new media provides a broader working platform for the management of college students. The traditional management platform for college students mainly include class meetings, school newspapers, publicity boards, symposiums, interviews, etc. These methods are limited by time and space and are relatively simple and often do not receive good educational effects. With the advent of new media, college students now have access to a platform for political and ideological education that was previously unattainable due to the constraints of time and geography. Relying on information technology, new media has the advantages of rich resources, strong interaction, and rapid dissemination compared with traditional media, creating a brand-new educational platform for college students and enabling student management workers to have a better understanding of students' needs channel. On this working platform, student management workers can carry out their work in a timely and comprehensive manner. Teachers and students can be friends on QQ and WeChat and engage on Weibo, allowing teachers to provide immediate and focused counsel to problems as they develop, influencing students' behavior, changing bad habits, and helping them progress. Student management staff use the new media platform to gather useful material to assist college students in growing up healthy and then broadcast it on the platform via text, video, audio, photos, and other means. According to statistics, there are 9 WeChat official accounts at various levels in a school, and each department also has its own WeChat official account. These official accounts have their own characteristics and push department news, student management, and student growth-related knowledge, which has a great impact on students
3. The new media has changed the working methods of the management of college students and promoted the communication between teachers and students. The new media has expanded the ideas of student management, integrated it into the management of students, and completely innovated the way of education. Before the new media era, an educational model centered on management educators, teaching materials, and classrooms was formed. To carry out managerial activities, managers primarily employed theoretical instillation and preaching. Students are in a submissive position and passively take information. Student administrators are frequently “arrogant” and require students to be managed. This concept has been dramatically transformed by the advent of new media. Workers in student management have modified their teaching techniques, included new media elements, and acted as guides in educational management activities. As a new working platform for college students' management job, new media tools like WeChat and Weibo have proved their merits. Students are ready to adopt a number of media formats in addition to conventional written language and text. For example, you can grasp the student's ideological dynamics by checking the students' QQ, Weibo, and WeChat. Send information through WeChat groups, forums, etc., and publish class dynamics, so that students can better participate in student management. The new media has provided more diverse and convenient working platforms for student management, changed the working methods of college students' management, and promoted the communication between teachers and students
4. The new media has formed a harmonious joint management environment. The so-called educational synergy is the comprehensive effect produced by the implementation of comprehensive education within a certain period of time and under certain conditions. This comprehensive effect is not the sum of the individual educational functions in comprehensive education, but a new educational force that is much larger than the individual educational functions. The student management work in colleges and universities can only form an educational synergy if they receive more support. New media can bind together the forces of education. First of all, parents do not need to go to school, but through new media platforms such as WeChat and blogs, they can easily understand the situation of students in school and give feedback on problems that arise, thus forming a harmonious educational joint force between the school and parents. This new educational synergy breaks through the limitations of the traditional education model, effectively realizes the cooperation between the school and the family, and maximizes the effect of student education. Second, new media enhances cohesion. To increase their popularity and competitiveness, numerous colleges and universities now display their style through multimedia platforms such as campus networks, WeChat public platforms, and post bars. Students enthusiastically participated in many events such as college style and contestant voting, which improved the school's external image. The style is displayed inside the school via the new media platform. Activities such as the selection of “the most beautiful counselor” and “the most American military instructor” conducted by a school have enhanced cohesion within a certain range, spread positive energy, and also played a supervisory role, which is conducive to the formation of a harmonious management environment
5. Crisis public relation events in the age of traditional media have few communication channels, slow speed, narrow scope, and passive acceptance of information by the audience. The new media has changed the communication relationship between the media and the audience and changed the traditional discourse environment. As soon as the material is provided through new media, it is easy for other media outlets to cite and distribute it. Information is being disseminated more quickly and with a broader breadth. The audience can express their own opinions, and positive public opinion and negative public opinion are tit-for-tat, which increases the difficulty of management. As university administrators, when dealing with crisis events, they should seize the right to speak as soon as possible, publish the real information of the event through new media, express their position, establish their authority in the online battlefield, guide students to correctly view emergencies, prevent students from obeying gossip and fake news, and avoid spreading the truth and triggering the escalation of the incident. Among the students of a certain school, there was a rumor that the dormitory would be adjusted on a large scale, which caused the discussion and anxiety of the majority of students. After learning about it, the student office swiftly posted official news via the WeChat public account, thereby stopping the spread of misinformation and restoring normal classroom management procedures

Through the above discussion, it can be seen that new media has been widely used in student management and has produced a very positive effect. Therefore, this paper constructs the application and effect evaluation indicators of new media in student management, as shown in Table 1. According to the corresponding input indicators, different levels of evaluation results can be obtained, which are divided into three levels.

### 3.3. Construction of the Evaluation Model

#### 3.3.1. Building the Model Framework

*(1) The Number of Layers of the BPNN Is Determined*. According to the basic theory above, this paper selects a three-layer network structure that can simulate any nonlinear mapping function, that is, a single hidden layer structure.

*(2) Determination of the Number of Input Layer Units*. According to the analysis of this paper, there are 12 indicators for the application and effect evaluation of new media in student management. Therefore, this paper sets the number of neurons in the input layer to 12.

*(3) Determination of the Number of Output Layer Units*. The purpose of constructing the BPNN model in this paper is to use relevant data to evaluate the effect of new media in student management. Therefore, the number of neurons in the output layer is 1, which is the effect level.

*(4) Calculation of the Total Number of Hidden Layer Units to Be Used*. Neural networks are better able to explain nonlinear mapping relationships when they include more hidden layer units. But excessive number of units will lower model training's efficiency. And the number of hidden layer units must be less than *N* − 1, where *N* is the number of training samples; otherwise, the built model cannot be generalized. This article is based on the following empirical formula:

(12) $$\begin{array}{c} h=\sqrt{m+n}+a, \end{array}$$

where *h* is the number of hidden layer units, *m* is the number of input layer units, *n* is the number of output layer units, and *a* is an integer in the interval [1, 9].

Start with 5 units and increase to 15 in turn to test the influence of different numbers of units on the model error, and select the number of optimal results as the number of middle-level units.

*(5) Determination of Activation Function*. In this paper, the tansig function is selected as the transfer function.

*(6) Determination of Other Parameters*. In this paper, the trainingdx algorithm is selected as the learning algorithm of the BPNN. The algorithm has a momentum project and can achieve self-adaptive adjustment. In this paper, the training accuracy is set to 1*e*^−5^; that is, the error level is below 0.00001. The learning rate setting range is (0.1, 0.9), and the learning rate is the convergence distance of the model when the correction calculation is performed. A smaller learning rate will reduce the training efficiency, and a larger learning rate is not conducive to finding the optimal weight matrix. Different learning rates are tested, and the settings are selected to make the model training the most effective learning rate. Other parameters are set according to the default parameters of MATLAB and do not change.

*(7) The Input Layer of the Final Constructed Model*. The input layer of the final constructed model framework is set with 12 units, representing 12 evaluation indicators. The output layer sets 1 unit, which represents the level of the effect. The number of units in the middle layer needs to be further confirmed in the empirical process. The transfer functions from the input layer unit to the middle layer unit and the middle layer unit to the output layer unit are all tansig functions, and the learning algorithm is the trainingdx algorithm.

#### 3.3.2. Simulation of the Model

*(1) Preprocessing of Sample Data*. Because the meanings of the data in each dimension in the indicator system are different, the units used are also very different. At the same time, the internal transfer of the model and the range of the activation function have limits. To construct a real mapping relationship, it is necessary to standardize the input range. The processed input will render the built model meaningless, and the input data needs to be processed. The processing method selected in this paper is normalization processing, which converts data of different dimensions into similar data structures.

*(2) BPNN Training*. In this paper, a trainable feedforward neural network is established through the newf function, and then, the trained model is saved.

*(3) Simulation Output*. Input the data of the sample to be tested into the trained BPNN, use the neural network model to calculate the predicted target value through the sim function, and then denormalize the predicted value to obtain the evaluation value. It is the evaluation value of the application and effect of new media on student management work.

## 4. Experiment and Analysis

### 4.1. Dataset and Simulation of BP Neural Network Model

All of the experimental data in this study comes from a university questionnaire survey, and the necessary big data is then arranged into a data set of 200 training sets and 40 test sets. The analog input command sets the relevant basic parameters. Since the predicted target value is based on the effect evaluation level, the output dimension is 1. The transfer function between each level adopts the tansig function. The result update frequency display is set to update the training results every 400 iterations. Due to the complexity of the sample data, in order to obtain more accurate training results, the number of iterations of the initial training is set to 5000 times. The training error target of the neural network is set to 1*e*^−5^, which is 0.00001. This error level can better reflect the simulation degree of the model and increase the reliability of the model. The gradient index used to detect the generalization ability of the model is set to l*e*^−6^. The generalization ability index is used to prevent the model from falling into a local minimum. The model stops running when the error reduction degree of the model training does not meet the defined generalization ability index. The trial-and-error method was used to conduct experiments with various numbers of middle-layer units, and the number of hidden layer units that made the model fit ideally was chosen as the number of middle-layer units in the BPNN model in this study. The relationship between the number of hidden layer units and the training error is shown in Figures 2–4. The number of nodes chosen for trials is 5, 7, 9, 11, 13, and 15. The training error reaches a minimum value when the number of hidden layer units is 9, as seen in the figure; hence, this study sets the number of hidden layer units to 9.

After trial-and-error experiments, it was found that too large a learning rate could easily make the neural network fall into a local minimum. When the learning rate is 0.4, the training error reaches the maximum value, and when the learning rate is 0.1, 0.2, 0.4, 0.5, and 0.7, the training error is very close, because the smaller the learning rate, the less likely the model will fall into the regional minimum value. Therefore, in order to obtain a better training effect, this paper sets the learning rate to 0.1.

The number of hidden layer units is set to 9 as described above, and the learning rate of the model is set to 0.1. After setting the relevant basic parameters, use the newff command to construct the BPNN, and set the neural network training function to the trainingdx function. After constructing the BPNN, use the command to run the MATLABR2020b program to train the model. The model's interpretation degree when the training is completed is *R* = 0.9999, according to the program's running results. The model's training accuracy is very good, and it has a strong ability to sample data, as can be observed. The trained evaluation model can better reflect the nonlinear mapping relationship between the input index and the output index of the sample data. Store the trained BPNN model. At this time, the BPNN model has been completed. You can input new sample data through the model to predict the evaluation level of the application effect of the new sample.

### 4.2. Experimental Results of the BP Model

Input the sample data to be tested, use the sim simulation function to input the data, output the evaluation result data through the BPNN model, and then denormalize the obtained predicted output value through the postmnmx inverse normalization function, and finally obtain the predicted output value to be tested. The BPNN model predicts the sample output value, which is the evaluation level of the application influence of new media in student management job. The results of this evaluation are shown in Table 2. The relevant data will be graded by school leaders and experts engaged in student management and compared with the experimental results obtained by the BPNN proposed in this paper. It can be seen from the experimental results that the error between the results obtained by the model proposed in this paper and the results evaluated by experts is very small, indicating that the BP model has superior performance.

## 5. Conclusion

New media has infiltrated every nook and cranny of people's lives, impacting every element of their existence. College students' thinking, study, living, and behavior habits have all been substantially influenced by the use of new media. The new media has opened up a plethora of possibilities for student affairs management, increased work efficiency, and reduced the gap between students and professors. Student affairs management is no longer limited by time and space, so that student affairs management workers can communicate with students, understand and mastering the situation of students, and also provide a convenient channel for students to communicate with student affairs management workers on an equal footing. The diversity of new media also provides a good platform for innovation in student affairs management. But at the same time, we cannot ignore the negative impact of new media on student affairs management. The intricate information provided by the new media dazzles the students who are not strong in screening ability and are easily confused and misled, which affects the growth and success of college students. As a result, it is critical to employ new media in student affairs administration. This study looks into and evaluates the current state of college students' use of new media, as well as the importance of incorporating new media into college student affairs management. The neural network is used to evaluate the effect of new media in student management, and the following work is finally completed: (1) This paper uses the literature analysis method to systematically study the development history, concept, connotation, and characteristics of new media and conduct a more in-depth study discussion. The research results of the current academic circles on the management of student affairs in the new media environment are summarized by referring to the literature. (2) The relevant BPNN technologies are introduced, followed by the construction of an assessment index for the application effect of new media on student management work and the design of an appropriate BP network structure. (3) Experiments are carried out with the self-designed data set. The experimental results show that the model designed in this paper has a small error and good performance.

## Figures and Tables

**Figure 1:** Neural network model diagram.

**Figure 2:** Training effect when *N* = 5 and *N* = 7.

**Figure 3:** Training effect when *N* = 9 and *N* = 11.

**Figure 4:** Training effect when *N* = 13 and *N* = 15.

**Table 1:** Application of new media in student management and evaluation indicators.

Index	Label
Accelerate the collection of student information	I_1_
Pay attention to students' mental health in a timely manner	I_2_
It is convenient to record and publish reward and punishment information	I_3_
Follow up on student employment in a timely manner	I_4_
Expanded work extension space for student administrators	I_5_
Provide a broader working platform for college students' management work	I_6_
Expanded the space of ideological and political education work	I_7_
Timely push college-related news	I_8_
Flexible and diverse educational methods	I_9_
Students are more willing to accept new media methods	I_10_
Integrate various educational forces	I_11_
Facilitate the organization of various new media-related events	I_12_

**Table 2:** Comparison of BP model output and expert evaluation results.

Number	1	2	3	4	5	6	7	8
Expert evaluation	0.75	0.77	0.85	0.88	0.92	0.63	0.71	0.66
Model output	0.73	0.76	0.85	0.90	0.92	0.61	0.73	0.65

## Data Availability

The datasets used during the current study are available from the corresponding author on reasonable request.
